# Chinese Medicine *Leptochloa chinensis* Inhibits the Malignant Behaviors of Renal Cell Carcinoma 786-O Cells by Regulating the mTOR Pathway

**DOI:** 10.1155/2021/5122380

**Published:** 2021-10-12

**Authors:** Yongshun Tan, Lingyun Li, Hongyue Liu, Jiadong Yu, Qijun Wang, Qiuju Lin

**Affiliations:** ^1^Department of Nephrology, Jinan City People's Hospital, Jinan People's Hospital Affiliated to Shandong First Medical University, Jinan 271199, Shandong Province, China; ^2^Department of Internal Medicine, Laishan Branch Hospital of Yantai Yuhuangding Hospital, Yantai, 264003, Shandong Province, China; ^3^Disinfection Supply Center, Affiliated Qingdao Central Hospital, Qingdao University, Qingdao, 266000, Shandong Province, China; ^4^Personnel Section, Zhangqiu District People's Hospital, Jinan, 250200, Shandong Province, China; ^5^Department of Otorhinolaryngology, Zhangqiu District People's Hospital, Jinan 250200, Shandong Province, China; ^6^Department of Oncology (II), Affiliated Qingdao Central Hospital, Qingdao University, Qingdao, 266000, Shandong Province, China

## Abstract

**Background:**

Renal cell carcinoma (RCC) is a common malignant tumor of the urinary system that seriously threatens human life and health. This study aims to explore the role of the traditional Chinese medicine *Leptochloa chinensis* in the pathogenesis of RCC. Meanwhile, this study also revealed the molecular biological mechanism of its antitumor activity.

**Methods:**

Human RCC 786-O cells were cultured in the RPMI-1640 medium, which contains different concentrations of *Leptochloa chinensis* (1,000, 3,000, and 9,000 *μ*g/ml). MTT and flow cytometry assays were used to detect the viability of 786-O cells. Transwell and wound healing assays were used to detect cell metastasis. The protein expression was observed by western blot analysis.

**Results:**

*Leptochloa* can inhibit cell proliferation and induce apoptosis in RCC 786-O cells. In addition, *Leptochloa* can weaken the migration and invasion of 786-O cells. More importantly, *Leptochloa* can block the mTOR pathway by inhibiting the protein expression of p-mTOR. Moreover, the high concentration of *Leptochloa chinensis* has a better inhibitory effect on 786-O cells.

**Conclusion:**

The traditional Chinese medicine *Leptochloa chinensis* inhibits the viability and metastasis of 786-O cells by blocking the mTOR pathway.

## 1. Introduction

Renal cell carcinoma (RCC) is a common malignant tumor of the urinary system, which seriously threatens human life and health [1]. RCC accounts for 2% to 3% of adult systemic malignant tumors, and its incidence is increasing at a rate of 2.5% per year [2]. In addition, RCC is relatively insidious and lacks sensitivity to radiotherapy and chemotherapy. Even with surgical treatment, there are still 20% to 40% of patients with postoperative invasion and distant metastasis [3]. Most RCC patients are already at an advanced stage when they are diagnosed. And the cause of death is related to tumor metastasis [4]. Therefore, seeking a new RCC treatment method is of great significance for prolonging the life of patients and improving the life quality of patients.

Isolating effective anticancer active ingredients from plants is one of the ways to find new anticancer drugs, and the antitumor effect of Chinese medicine has been recognized [5]. Previous studies have confirmed that the antitumor effects of some Chinese medicines have ideal effects [6, 7]. *Leptochloa chinensis*, also known as “Pusa bean, Qianliangjin,” is the dry mature seed of *Euphorbia lathyris* L. [8]. As early as the 1920s, foreign scholars conducted relevant research on the Chinese medicine *Leptochloa chinensis* [9]. At present, it has also been found that *Leptochloa chinensis* has pharmacological activity on a variety of tumor cells. It has been reported that *Leptochloa chinensis* is used to treat esophageal cancer [10], skin tumors [11], and acute lymphocytic leukemia [12], with good curative effects.

It has been shown that the mTOR pathway is closely related to tumor proliferation, invasion, and metastasis [13]. Blocking the PI3K/AKT/mTOR signaling pathway can inhibit tumor cell proliferation and metastasis and even induce cell apoptosis [14]. Li et al. found that plumbagin can block the PI3K/AKT/mTOR signaling pathway, leading to lung cancer cell apoptosis [15]. However, the specific anticancer mechanism between *Leptochloa chinensis* and mTOR signaling pathway is still unclear.

Therefore, this study explored whether *Leptochloa chinensis* can inhibit the proliferation, invasion, and migration of 786-O RCC cells. The anticancer mechanism of *Leptochloa chinensis* was also investigated in 86-O RCC cells. This study aims to provide more theoretical basis for the antitumor of Chinese medicine.

## 2. Materials and Methods

### 2.1. Preparation of Lathyrol

The experimental drug of lathyrol was purchased from Sichuan Weikeqi Biological Technology Co., Ltd., with a purity of 99% (no. 20190023, 20 mg/bottle). The drug was dissolved in 200 *μ*l dimethyl sulfoxide (DMSO), and then PBS was added to 2 ml. RPMI-1640 culture medium containing 10% fetal bovine serum (FBS) was used to dilute lathyrol to the experimental design concentration (0, 1000, 3000, and 9000 *μ*g/ml).

### 2.2. Cell Culture

First, 786-O RCC cells were divided into 4 groups (one of which is a blank control). After digesting the cells with 0.25% trypsin, a single cell suspension was prepared with the RPMI-1640 medium containing 10% FBS. The cell concentration was adjusted to 6 × 10^5^ cells/ml, and the cells were seeded in a 96-well plate with 100 *μ*l per well. After culturing in an incubator with 5% CO_2_ at 37°C for 24 h, the medium was added to each well to make up to 100 *μ*l.

### 2.3. MTT Assay

Four groups of 786-O RCC cells were cultured with 0, 1000, 3000, and 9000 *μ*g/ml lathyrol. The dose was added once a day for 5 consecutive days. 24 h after the last dose, 10 *μ*l of 5 mg/ml MTT solution was added to each well. After incubating for 4 h, the supernatant was discarded. 110 *μ*l DMSO was added to each well, and the cells were incubated for 10 min at room temperature. The absorbance value (OD value) was measured at 490 nm by the enzyme-linked immunosorbent assay. Inhibition rate (%) = (OD value of the blank group − OD value of the experimental group)/OD value of the blank group × 100%.

### 2.4. Flow Cytometric Analysis

786-O RCC cells (6 × 10^5^ cells/ml) were evenly added into a 6-well cell culture plate. Then, it was placed in a constant temperature cell incubator for 24 h. After adherence, different concentrations of lathyrol (0, 1000, 3000, and 9000 *μ*g/ml) were added to the cells. After regular incubation for 24 h, they were digested with 5% trypsin without EDTA. Next, 500 *μ*l buffer, 5 *μ*l annexin V, and 5 *μ*l PI were added to the cells in sequence. After 30 minutes of reaction in the dark at room temperature, the flow cytometer detected cell apoptosis within 1 h. The results obtained were analyzed with FlowJo software.

### 2.5. Wound Healing Assay

786-O RCC cells were immediately seeded into a 6-well plate with a density of 6 × 10^5^ per well. After the cells adhered, the cells were starved with a serum-free medium for 6 h. Next, a 200 *μ*l pipette tip was used to make a “1”-shaped scratch in the direction perpendicular to the 6-well plate. Different concentrations (0, 1000, 3000, and 9000 *μ*g/ml) of lathyrol were then added. After 24 h, the width of the scratch was observed under an inverted microscope. Cell migration rate (%) = (0 h scratch spacing − 24 h scratch spacing)/0 h scratch spacing × 100%.

### 2.6. Transwell Assay

Transwell chamber assay was used to detect the invasion ability of 786-O RCC cells *in vitro*. First, 500 *μ*l of the RPMI-1640 cell culture medium without FBS was added to the bottom well. The upper chamber was added with 100 *μ*l cell suspension, Matrigel (BD Biosciences), and different concentrations of lathyrol. Then, the cells were placed in a cell incubator with saturated humidity at 37°C with 5% CO_2_ for 48 h. Next, the cells were fixed with 4% paraformaldehyde for 30 min and then stained with 0.1% crystal violet for 20 min. The invasive cells were observed and counted under a microscope.

### 2.7. Western Blot Assay

RIPA Lysis Buffer (Beyotime, Shanghai, China) was used to extract total protein from 786-O RCC after treatment with lathyrol. The BCA kit was used to detect protein concentration. Then, 50 *μ*g protein was used for the SDS-PAGE experiment. The protein sample was transferred to the PVDF membrane and blocked with 5% skimmed milk at 37°C for 1.5 h. The membrane was washed 5 times with TBST. The protein samples were then incubated with Bax, Bcl-2, mTOR, and p-mTOR primary antibodies in a refrigerator at 4°C overnight. Next, the protein was incubated with secondary antibodies for 2 h at room temperature. Subsequently, ECL exposure and development were performed in the ChemiDoc imaging system. *β*-Actin was used as an internal control. Quantity One 4.52 analysis software was used to measure the gray value of the bands. The relative expression of the target protein (IOD) = the gray value of the target protein/the gray value of the internal reference *β*-actin.

### 2.8. Statistical Analysis

Statistical analysis was performed using SPSS 24.0 software. The data are shown as mean ± SD. All experiments are repeated three times. The differences were analyzed by Student's *t*-test or one-way ANOVA followed by Tukey's post hoc test. *P* < 0.05 indicates a significant difference.

## 3. Results

### 3.1. *Leptochloa* Inhibits the Growth of RCC 786-O Cells

First, the effect of *Leptochloa* on the viability of RCC cells was investigated in 786-O cells. MTT assay showed that *Leptochloa* can inhibit the proliferation of 786-O cells (*P* < 0.05, Figure 1, Table 1). In addition, we also found that the inhibitory effect of *Leptochloa* on the proliferation of 786-O cells was enhanced with the increase of *Leptochloa* concentration. 9000 *μ*g/ml *Leptochloa* has the highest inhibitory effect, with a growth inhibition rate of 76.03% (*P* < 0.01, Figure 1, Table 1). These results indicate that high concentrations of *Leptochloa* can significantly inhibit cell proliferation in RCC.

### 3.2. *Leptochloa* Promotes the Apoptosis of RCC 786-O Cells

Compared with the blank group, the apoptotic rate of 786-O cells increased after the treatment with *Leptochloa*. The higher the concentration of *Leptochloa*, the higher the apoptosis rate of 786-O cells (*P* < 0.05, Figure 2(a)). The apoptotic rate of 786-O cells reached the highest at 9000 *μ*g/ml *Leptochloa*, which was 53.06% (Figure 2(a)). In addition, compared with the blank group, the expression of proapoptotic protein Bax was significantly increased after 786-O cells were treated with *Leptochloa*, while the expression of antiapoptotic protein Bcl-2 was significantly decreased (*P* < 0.05, Figure 2(b)). These results indicate that *Leptochloa* can induce apoptosis of 786-O cells.

### 3.3. *Leptochloa* Inhibits the Metastasis of RCC 786-O Cells

To investigate whether *Leptochloa* affects the metastasis of 786-O cells, wound healing assay and tanswell assay were performed. Wound healing assay showed that the migration distance of 786-O cells treated with *Leptochloa* was significantly shorter compared with the blank group (*P* < 0.05, Figure 3(a)). Among them, the 9000 *μ*g/ml group had the shortest migration distance (Figure 3(a)). Transwell assay showed that the number of invasive 786-O cells treated with *Leptochloa* was significantly reduced compared with the blank group (*P* < 0.05, Figure 3(b)). The higher the concentration of *Leptochloa*, the smaller the number of cells invaded (Figure 3(b)). These results indicate that *Leptochloa* can weaken the migration and invasion ability of 786-O cells.

### 3.4. *Leptochloa* Regulates the mTOR Pathway in RCC 786-O Cells

Western blot assay showed that, after treating 786-O cells with different concentrations of *Leptochloa* (1000, 3000, and 9000 *μ*g/mL), the mTOR protein expression of each drug group was not statistically different from that of the blank group (*P* > 0.05, Figure 4). However, the expression of p-mTOR protein was decreased with increasing concentration of *Leptochloa* (*P* < 0.05, Figure 4). The above results indicate that *Leptochloa* can block the mTOR pathway by inhibiting the protein expression of p-mTOR.

## 4. Discussion

RCC ranks second in malignant tumors of the urinary system, accounting for 3% of all solid tumors. With the continuous advancement of modern diagnostic technology, clinical cases of RCC have gradually increased [16]. However, 50% of RCC patients will metastasize after surgery. These patients require biological and immunotherapy [17]. Although great progress has been made in recent years, the overall effective rate of RCC is still low [18]. Therefore, people strive to explore the biological characteristics of RCC and possible effective treatments of Chinese medicine from the molecular biology level to significantly improve the prognosis of RCC.

In recent years, previous studies have found that *Leptochloa chinensis* has an inhibitory effect on a variety of tumor cells. For example, it was discovered earlier that *Leptochloa chinensis* had obvious anti-mouse ascites sarcoma cell activity [19]. This study found that *Leptochloa chinensis* had an inhibitory effect on the proliferation of 786-O cells. And the higher the concentration of *Leptochloa chinensis*, the stronger the anticancer effect. Choene et al. found that, with the increase of *Leptochloa chinensis* concentration, the number of human renal cancer cells in the G0 phase increases [20]. This also shows that *Leptochloa chinensis* has an inhibitory effect on the growth of human RCC cells. In addition, cell invasion and migration are other important factors that affect the prognosis and the main reason for the failure of tumor treatment [21]. In this study, transwell and wound healing assays showed that *Leptochloa chinensis* can effectively inhibit cell migration and invasion in RCC cells. Yang et al. also showed that *Leptochloa chinensis* suppressed the invasion and metastasis of human lung cancer A549 cells [22], similar to the results of this study. These results indicate that traditional Chinese medicine *Leptochloa chinensis* can inhibit the progression of RCC.

Recent studies have shown that the PI3K/AKT/mTOR signaling pathway is widely present in a variety of cells and is involved in the regulation of cell proliferation, apoptosis, invasion, metastasis, and angiogenesis [23]. The dysregulation of the PI3K/AKT/mTOR signaling pathway is related to the occurrence and development of many human cancers. Han et al. found that L-securinine promoted human acute myeloid leukemia cell HL-60 apoptosis through the PI3K/AKT/mTOR pathway [24]. In addition, Li et al. showed that traditional Chinese medicine curcumin downregulated mTOR to promote autophagy and apoptosis of lung cancer A549 cells [15]. These studies indicate that the antitumor effect of traditional Chinese medicine *Leptochloa chinensis* may also be achieved by inhibiting the protein expression of mTOR or p-mTOR. As we predicted, *Leptochloa chinensis* can significantly downregulate the expression of p-mTOR, but has no significant effect on the expression of mTOR. The results indicate that *Leptochloa chinensis* may inhibit cell proliferation, invasion, and migration by regulating the expression of p-mTOR.

## 5. Conclusion

In summary, *Leptochloa chinensis* can inhibit cell viability, invasion, and migration of 786-O cells. And the higher the concentration of *Leptochloa chinensis*, the stronger its inhibitory effect on RCC. We also found that *Leptochloa chinensis* exerts its anticancer effect in RCC by preventing the activation of mTOR phosphorylation. These results provide more theoretical basis for Chinese medicines to fight cancer. As for the other antitumor mechanisms of *Leptochloa chinensis*, further research is needed.

## Figures and Tables

**Figure 1:** *Leptochloa* inhibits the growth of RCC 786-O cells. Cell proliferation was detected in 786-O cells treated with different concentrations of lathyrol (0, 1000, 3000, and 9000 *μ*g/ml). ^*∗*^*P* < 0.05 and ^*∗∗*^*P* < 0.01.

**Figure 2:** *Leptochloa* promotes the apoptosis of RCC 786-O cells. (a) Cell apoptosis was detected in 786-O cells treated with different concentrations of lathyrol (0, 1000, 3000, and 9000 *μ*g/ml). (b) The protein expression of Bax and Bcl-2 was measured in 786-O cells treated with different concentrations of lathyrol (0, 1000, 3000, and 9000 *μ*g/ml). ^*∗*^*P* < 0.05 and ^*∗∗*^*P* < 0.01.

**Figure 3:** *Leptochloa* inhibits the metastasis of RCC 786-O cells. (a) Cell migration was detected by the wound healing assay in 786-O cells treated with different concentrations of lathyrol (0, 1000, 3000, and 9000 *μ*g/ml). (b) Cell invasion was detected by the transwell assay in 786-O cells treated with different concentrations of lathyrol (0, 1000, 3000, and 9000 *μ*g/ml). ^*∗*^*P* < 0.05 and ^*∗∗*^*P* < 0.01.

**Figure 4:** *Leptochloa* regulates the mTOR pathway in RCC 786-O cells. The protein expression of mTOR and p-mTOR was measured in 786-O cells treated with different concentrations of lathyrol (0, 1000, 3000, and 9000 *μ*g/ml). ^*∗*^*P* < 0.05 and ^*∗∗*^*P* < 0.01.

**Table 1:** The inhibitory effect of different concentrations of *Leptochloa* on the proliferation of 786-O cells.

*Leptochloa* concentrations	OD value	Inhibition rate (%)	*P* value
0 (blank group)	0.999	—	—
1000 *μ*g/ml	0.463	53.65	0.018^*∗*^
3000 *μ*g/ml	0.337	66.27	0.012^*∗*^
9000 *μ*g/ml	0.241	75.88	0.008^*∗∗*^

^*∗*^ *P* < 0.05 and ^*∗∗*^*P* < 0.01.

## Data Availability

The datasets used during the present study are available from the corresponding author upon reasonable request.
